# Analysis on the Effects of CT- and Ultrasound-Guided Percutaneous Transthoracic Needle Biopsy Combined with Serum CA125 and CEA on the Diagnosis of Lung Cancer

This article has been retracted.

**DOI:** 10.1155/2022/2289432

**Published:** 2022-01-07

**Authors:** Zhaoyin Wang, Jinbiao Huang, Minke Wang, Weixu Bi, Tianbing Fan

**Affiliations:** ^1^Department of Radiology, Taizhou Hospital of Zhejiang Province Affiliated to Wenzhou Medical University, Taizhou 317000, Zhejiang, China; ^2^Department of Ultrasound, Taizhou Hospital of Zhejiang Province Affiliated to Wenzhou Medical University, Taizhou 317000, Zhejiang, China

## Abstract

The number of patients with lung cancer is difficultly diagnosed in the early stage. The purpose of the study was to investigate the effects of CT- and ultrasound-guided percutaneous transthoracic needle biopsy combined with serum CA125 and CEA on the diagnosis of lung cancer. 120 patients with suspected lung cancer admitted to our hospital from January 2019 to January 2020 were selected and divided into an ultrasound group (*n* = 60) and CT group (*n* = 60), according to different percutaneous transthoracic needle biopsy modalities. All patients received serum tumor markers detection, so as to compare the CT- and ultrasound-guided percutaneous transthoracic needle biopsy results and pathology results, levels of serum tumor markers among all patients and the patients with different lung cancer types, and diagnostic efficacy of tumor markers, as well as complication rate (CR) in patients. The sensitivity and specificity of ultrasound-guided percutaneous transthoracic needle biopsy were 0.880 and 0.800, respectively, while those of CT-guided percutaneous transthoracic needle biopsy were 0.909 and 0.625, respectively; the CA125 and CEA levels in the lung cancer group were higher than those in the benign group (*P* < 0.001); the CA125 and CEA levels of the patients with adenocarcinoma were higher than those with squamous carcinoma, and the CEA levels of the patients with small-cell carcinoma were lower than those with adenocarcinoma (*P* < 0.05); the sensitivity, specificity, and Youden indexes of CA125 were 0.638, 0.833, and 0.471, respectively, while those of CEA were 0.766, 0.778, and 0.544, respectively; there were no significant differences in CR between the two groups (*P* > 0.05). CT- and ultrasound-guided percutaneous transthoracic needle biopsy is a safe and feasible diagnostic modality for lung cancer, and its combination with serum CA125 and CEA can significantly improve the accuracy of the detection results, which is worthy of promotion and application in clinical practice.

## 1. Introduction

The number of patients with lung cancer has soared across the world in recent years, and when diagnosed, the patients have entered the advanced stage of the disease, severely hindering treatment progress [1–3] and resulting in the death rate staying at a high level. More research on the diagnosis of lung cancer must be intensified in clinical practice to improve the diagnosis rate. CT-guided percutaneous transthoracic needle biopsy, with high safety, can avoid some damage to patients' vessels, but this examination modality may cause complications in patients under the influence of multiple risk factors, thus ultimately leading to unsatisfactory application outcomes. Ultrasound-guided percutaneous transthoracic needle biopsy can protect patients from suffering from complications such as hemoptysis, but its precision is suboptimal. Consequently, both examination modalities have certain limitations [4–7]. In addition to the two examination modalities mentioned above, serum tumor markers' detection has also become a hot spot of clinical research recently, though with the drawbacks of difficult localization, which can be fully used to carry out joint examinations with percutaneous transthoracic needle biopsy, increasing the accuracy of location and improving diagnostic rate [8–11]. Ultrasound- and CT-guided percutaneous transthoracic needle biopsy modalities are very common [12–15], with the former characterized by being minimally invasive and safe. Generally, the accuracy of imageological examination in judging lung cancer is limited, while serum tumor markers can enhance physicians' knowledge, such as lung cancer cell differentiation, and are of great importance in judging patients' lung cancer conditions and classification [15–19]. Generally, the accuracy of imageological examination in judging lung cancer is limited, while serum tumor markers can enhance physicians' knowledge, such as lung cancer cell differentiation, and are of great importance in judging patients' lung cancer conditions and classification [15–19]. Based on this, in our study, with the purpose of investigating to explore the effects of CT- and ultrasound-guided percutaneous transthoracic needle biopsy combined with serum CA125 and CEA on the diagnosis of lung cancer, 120 patients with suspected lung cancer admitted to our hospital from January 2019 to January 2020 were selected as the study subjects, and the study results are summarized as follows.

## 2. Materials and Methods

### 2.1. General Information

120 patients with suspected lung cancer admitted to our hospital from January 2019 to January 2020 were selected and divided into an ultrasound group (*n* = 60) and CT group (*n* = 60), according to different modalities of percutaneous transthoracic needle biopsy. There were no significant differences in the general information between the two groups (*P* > 0.05), and the patients and their family members signed the informed consent, as shown in Table 1.

### 2.2. Inclusion Criteria

(1) Patients were diagnosed with space-occupying lesions in their lungs by imageological examination. (2) Patients underwent surgical treatment and obtained pathological results. (3) This study was approved by the hospital ethics committee.

### 2.3. Exclusion Criteria

(1) Patients had mental disorders and could not communicate with others. (2) Patients had other organic diseases. (3) Patients had coronary heart disease, arrhythmia, and coagulation disorders.

### 2.4. Methods

All patients received serum tumor marker detection. In the ultrasound group, the patients underwent ultrasound-guided percutaneous transthoracic needle biopsy, while the CT group patients were given CT-guided percutaneous transthoracic needle biopsy, and the specific methods were as follows.

#### 2.4.1. Serum Tumor Marker Detection

Patients' fasting venous blood samples were collected in the morning, and the serum was isolated after self-coagulation and stored in a freezer at −25°C for detection within 3 days. The CA125 and CEA levels were measured by the electrochemiluminescence immunoassay (Cobase 411 electrochemiluminescence instrument with original auxiliary reagents; CFDA (I) 20113402843).

#### 2.4.2. Ultrasound-Guided Percutaneous Transthoracic Needle Biopsy

After the location of lung lesions was clarified by chest CT in patients, an ultrasound probe (GE Medical; Voluson P6 color ultrasonic device; CFDA 20152062178) was adopted to examine the affected tissues and their structure to determine the needle entry position. Then, the puncture sites were sterilized and given local anesthesia, and the puncture angle, depth, etc., were all checked before an ultrasound-guided percutaneous transthoracic needle biopsy. After that, the biopsy tissues were fixed with 10% formaldehyde solution (Shanghai Solvent Factory; State Food and Drug Administration approval number: H31020858) for detection.

#### 2.4.3. CT-Guided Percutaneous Transthoracic Needle Biopsy

The location of the lesions in patients' lungs was clarified according to the chest CT, and the patients were asked to take appropriate positions. The lesions were scanned with 3 mm in each layer by using a CT scanner (Philips brilliance16-slice Spiral CT instrument; CFDA (I) 20093300931), and metal bar localizers were placed in the corresponding body surface sites. After that, the scanning continued, to determine the appropriate puncture sites, and the puncture angle, depth, etc., were calculated by measuring before the puncture sites were disinfected and given local anesthesia. Then, a biopsy gun (Guangzhou Qihe Medical Instrument Co., Ltd.; Guangdong Food and Drug Certified No. 20181153) was used after the puncture needles were confirmed inside the mass by scanning, and the biopsy tissues were fixed with 10% formaldehyde solution before detection.

### 2.5. Observation Indexes

1. CT- and ultrasound-guided percutaneous transthoracic needle biopsy results and pathology results were compared to calculate the sensitivity and specificity of the two diagnostic methods
2. Serum tumor markers levels: the patients were divided into the lung cancer group and the benign group, according to their pathological findings, and the serum CA 125 and CEA levels were compared between the two groups
3. Serum tumor markers levels in patients with different lung cancer types: the serum CA125 and CEA levels of the patients with adenocarcinoma, squamous carcinoma, and small-cell carcinoma were compared
4. Diagnostic efficacy of tumor markers: the sensitivity, specificity, and Youden indexes of serum CA125 and CEA were compared, and the value of Youden indexes close to 1 indicated higher authenticity and better diagnosis [20–22]
5. CR: the cases of complications including pneumothorax, hemorrhage, and hemoptysis were recorded

### 2.6. Statistical Treatment

The selected data processing software for this study was SPSS20.0, and the software selected to draw the pictures of the data was GraphPad Prism 7 (GraphPad Software, San Diego, USA). Measurement data were tested by the *t*-test, and enumeration data were tested by the *X*^2^ test and normality test. The differences had statistical significance when *P* < 0.05.

## 3. Results

### 3.1. Comparison of CT- and Ultrasound-Guided Percutaneous Transthoracic Needle Biopsy Results and Pathology Results

The sensitivity and specificity of CT- and ultrasound-guided percutaneous transthoracic needle biopsy are shown in Table 2.

### 3.2. Comparison of the Levels of Serum Tumor Markers

The CA125 and CEA levels in the lung cancer group were higher than those in the benign group (*P* < 0.001), as shown in Figures 1 and 2.

### 3.3. Comparison of Serum Tumor Marker Levels in Patients with Different Lung Cancer Types

The CA125 and CEA levels of the patients with adenocarcinoma were higher than those with squamous carcinoma, and the CEA levels of the patients with small-cell carcinoma were lower than those with adenocarcinoma (*P* < 0.05), as shown in Table 3.

### 3.4. Comparison of the Diagnostic Efficacy of Tumor Markers

The diagnostic efficacy of CA125 and CEA is shown in Table 4.

### 3.5. Comparison of CR between the Two Groups

There were no significant differences in CR between the two groups (*P* > 0.05), as shown in Figure 3.

## 4. Discussion

Nowadays, lung cancer has become a leading cause of death, and early diagnosis and treatment can reduce patients' case fatality rate and ensure their physical health. Until now, there are many means in the diagnosis of lung cancer in patients, but each has its limitations; in comparison, percutaneous transthoracic needle biopsy is a more ideal examination method, with significant advantages of high safety and reliability, which has achieved wide application in clinical practice. Ultrasound- and CT-guided percutaneous transthoracic needle biopsy modalities are very common [12–15], with the former characterized by being minimally invasive and safe. This study showed the sensitivity and specificity of the ultrasound-guided percutaneous transthoracic needle biopsy were 0.880 and 0.800, respectively, which are close to the results of general studies in the academic community, and the factors affecting its precision mainly include patients' body conditions. For example, inflated lung can hinder the detection. CT-guided percutaneous transthoracic needle biopsy can localize tiny tissues and can compensate for the exploration limitations in the ultrasound-guided one. This study revealed that the sensitivity and specificity of CT-guided percutaneous transthoracic needle biopsy were 0.909 and 0.625, indicating that CT-guided percutaneous transthoracic needle biopsy also has good application value, but this modality takes patients a great expense and has severe radiation, so the selection of examination modalities should be based on patients' own conditions.

In addition to a percutaneous transthoracic needle biopsy, serum tumor markers detection is also a routine diagnostic modality for lung cancer. Generally, the accuracy of imageological examination in judging lung cancer is limited, while serum tumor markers can enhance physicians' knowledge, such as lung cancer cell differentiation, and are of great importance in judging patients' lung cancer conditions and classification [15–19]. In this study, the CA125 and CEA levels in the lung cancer group were higher than those in the benign group (*P* < 0.001), and the CA125 and CEA levels of the patients with adenocarcinoma were higher than those with squamous carcinoma, and the CEA levels of the patients with small-cell carcinoma were lower than those with adenocarcinoma (*P* < 0.05), suggesting that tumor markers can effectively diagnose lung cancer, among which CEA has a high sensitivity for adenocarcinoma. CA125 is also a major marker of adenocarcinoma, and the reason why CA125 levels increase in lung cancer patients is that the CA125 antigen inside patients' bodies is stimulated and then constantly released and finally enters the blood through autonomous absorption, elevating CA125 levels.

## 5. Conclusions

In this study, the sensitivity, specificity, and Youden indexes of CA125 were 0.638, 0.833, and 0.471, respectively, while those of CEA were 0.766, 0.778, and 0.544, confirming that CEA and CA with high clinical application value can combine with percutaneous transthoracic needle biopsy to further improve the diagnosis rate of lung cancer. The scholar Wanda Lawrence has pointed out in his study that the Youden indexes of CA125 and CEA are 0.475 and 0.544, respectively [23], and their combination with percutaneous transthoracic needle biopsy can increase the diagnosis rate of lung cancer in patients, which is in line with the conclusions drawn in our study, indicating that the two tumor markers can be applied in the clinical diagnosis of lung cancer.

Moreover, our study results also found that CR in both groups was low, and there were no significant differences between groups (*P* > 0.05), confirming that ultrasound- and CT-guided percutaneous transthoracic needle biopsy have high safety and feasibility, which can be applied widely in clinical treatment.

In conclusion, CT- and ultrasound-guided percutaneous transthoracic needle biopsy combined with serum CA125 and CEA, with high application value, can further improve the diagnosis rate of lung cancer in patients, which is worthy of application and promotion in clinical practice.

## Figures and Tables

**Figure 1:** Comparison of CA125 levels between the lung cancer and the benign group ($\bar{x}$ ± *s*, U/ml). The abscissa represents the lung cancer group (*n* = 94) and benign group (*n* = 26), while the ordinate represents the CA125 level (U/ml). The CA125 levels were (34.50 ± 5.23) U/ml in the lung cancer group and (16.68 ± 7.85) U/ml in the benign group. ^*∗*^*P* < 0.001.

**Figure 2:** Comparison of CEA levels between the lung cancer and the benign group ($\bar{x}$ ±*s*, ng/ml). The abscissa represents the lung cancer group (*n* = 94) and benign group (*n* = 26), while the ordinate represents the CEA level (ng/ml). The CEA levels were (14.05 ± 2.89) ng/ml in the lung cancer group and (3.56 ± 0.89) ng/ml in the benign group. ^*∗*^*P* < 0.001.

**Figure 3:** Comparison of CR between the two groups. The black area represents pneumothorax, the dark gray area represents hemorrhage, the light gray area represents hemoptysis, and the yellow area represents no complications. The left figure represents the ultrasound group, while the right figure represents the CT group. The number of the patients with pneumothorax was 2 in the ultrasound group and 3 in the CT group. The number of the patients with hemorrhage was 1 in the ultrasound group and 2 in the CT group. The number of the patients with hemoptysis was 3 in the ultrasound group and 3 in the CT group. The number of the patients with no complications was 54 in the ultrasound group and 52 in the CT group.

**Table 1:** Comparison of general information between the two groups.

Group	Cases	Gender (male/female)		Average age **(years)**
Ultrasound group	60	35	25	45.21 ± 5.65
**CT group**	60	34	26	45.32 ± 5.78
**t/X** ^**2**^			0.034	0.105
*P*			0.853	0.916

**Table 2:** Comparison of CT- and ultrasound-guided percutaneous transthoracic needle biopsy results and pathology results.

Diagnostic methods		Pathology results		Sensitivity	Specificity
		Malignant	Benign		
Ultrasound (*n* = 60)	Malignant	44	2	0.880	0.800
	Benign	6	8		

**CT** (*n* = 60)	Malignant	40	6	0.909	0.625
	Benign	4	10		

**Table 3:** Comparison of serum tumor marker levels in patients with different lung cancer types.

Group	Cases	CA125 (U/ml)	CEA (ng/ml)
Squamous carcinoma	40	30.12 ± 15.68	35.62 ± 15.78
Adenocarcinoma	34	38.56 ± 15.45^*∗*^	43.89 ± 16.41^*∗*^
Small-cell carcinoma	20	34.10 ± 15.46	30.10 ± 13.56^#^

^*∗*^The comparison with the squamous carcinoma group, *P* < 0.05; ^#^the comparison with the adenocarcinoma group, *P* < 0.05.

**Table 4:** Comparison of the diagnostic efficacy of tumor markers.

Diagnostic methods	Sensitivity	Specificity	Youden index
CA125	0.638	0.833	0.471
CEA	0.766	0.778	0.544

## Data Availability

The datasets used and/or analyzed during the current study are available from the corresponding author on reasonable request.
